The article "Advanced Cognitive Algorithm for Biomedical Data Processing: COVID-19 Pattern Recognition as a Case Study" was retracted in 2023. Reasons: signs of a paper mill; suspected computer-generated content; unreliable results or conclusions; concerns about the data.

# Advanced Cognitive Algorithm for Biomedical Data Processing: COVID-19 Pattern Recognition as a Case Study

**DOI:** 10.1155/2022/1773259

**Published:** 2022-03-22

**Authors:** Mohamed Elhoseny, Zahraa Tarek, Ibrahim M. EL-Hasnony

**Affiliations:** ^1^College of Computing and Informatics, University of Sharjah, Sharjah, UAE; ^2^Faculty of Computers and Information, Mansoura University, Mansoura, Egypt

## Abstract

Automated disease prediction has now become a key concern in medical research due to exponential population growth. The automated disease identification framework aids physicians in diagnosing disease, which delivers accurate disease prediction that provides rapid outcomes and decreases the mortality rate. The spread of Coronavirus disease 2019 (COVID-19) has a significant effect on public health and the everyday lives of individuals currently residing in more than 100 nations. Despite effective attempts to reach an appropriate trend to forecast COVID-19, the origin and mutation of the virus is a crucial obstacle in the diagnosis of the detected cases. Even so, the development of a model to forecast COVID-19 from chest X-ray (CXR) and computerized tomography (CT) images with the correct decision is critical to assist with intelligent detection. In this paper, a proposed hybrid model of the artificial neural network (ANN) with parameters optimization by the butterfly optimization algorithm has been introduced. The proposed model was compared with the pretrained AlexNet, GoogLeNet, and the SVM to identify the publicly accessible COVID-19 chest X-ray and CT images. There were six datasets for the examinations: three datasets with X-ray pictures and three with CT images. The experimental results approved the superiority of the proposed model for cognitive COVID-19 pattern recognition with average accuracy 90.48, 81.09, 86.76, and 84.97% for the proposed model, support vector machine (SVM), AlexNet, and GoogLeNet, respectively.

## 1. Introduction

The first infections of coronavirus disease in December 2019 (COVID-19) were recorded in a significant city in China called Wuhan. COVID-19 originates from the SARS-CoV-2 virus and is now mono of the main issues in the world. Thousands of deaths and confirmed cases worldwide are outlined from COVID-19. The high number of infections is indicative of the rapid spread between people population.

The signs of COVID-19 familiar to date involve high temperature, sore throat, cough, migraine, vomiting, muscle aches, and other symptoms. Another critical factor is the early diagnosis of COVID-19 can be mirrored in early remedy. This pandemic does not only affect the countries health, but the effects of COVID-19 are also significant (e.g., economic and psychic) [1]. So, COVID-19 is an epidemic with a wide range of threats that should be subtended. Based on the above facts, artificial intelligence models are needed to allow the recognition of this deadly virus in the reasonable time.

The article "Advanced Cognitive Algorithm for Biomedical Data Processing: COVID-19 Pattern Recognition as a Case Study" was retracted in 2023. Reasons: signs of a paper mill; suspected computer-generated content; unreliable results or conclusions; concerns about the data.

On the other side, the utilization of medical photographs to detect diseases has expanded in recent years. To identify infection caused by disease, various machine vision, and image recognition techniques provide accurate and rapid results. The findings, however, must be checked by a specialist. In this manner, medical image recognition techniques can be applied as an initial diagnostic tool that hints about a potential illness.

Artificial Intelligence (AI), with countless promising reports, has been widely used in our daily operations for managing the COVID-19 epidemic. AI approaches, including deep learning, have been applied for medical imaging to manipulate and analyze data to help clinicians and radiologists for enhancing diagnostic efficiency. Similarly, a host of research based on the automated identification of COVID-19 using deep learning algorithms have been applied [2]. AI approaches could also show their high efficiency in encouraging administrators to make smarter decisions on controlling viruses when thousands of health data are gathered by exchanging data between and across innovative countries using the recommended standards [3].

A variety of experiments have been presented to categorize COVID-19 from CT scan or X-ray images using various methodologies, such as ResNet-50, CNNs with Support Vector Machine (SVM), AlexNet, SqueezeNet, DenseNet201, VGG19, DRE-Net, and GoogLeNet. In common, it is often popular to extract various features from images and construct a collection containing details about the extracted features.

The significant contributions of this paper are summarized into three folds. In the first fold, an examination of the state-of-the-art solutions of artificial intelligence to tackle COVID-19 has been presented. As, this study introduces a systematic analysis for the most recent trials on COVID-19 using machine learning and deep learning methods; the used datasets, the tasks, and the outcomes of these trials are listed. Second, a comparative study for two pretrained models of the Convolutional Neural Network (CNN), namely, AlexNet, GoogLeNet, and Support Vector Machine (SVM) has been discussed. Also, the suggested approach is presented based on two categories of medical images: computerized tomography (CT) scanning and X-ray images. Third, a model based on the artificial neural network and the butterfly optimization algorithm for parameter adaption has been proposed.

The article "Advanced Cognitive Algorithm for Biomedical Data Processing: COVID-19 Pattern Recognition as a Case Study" was retracted in 2023. Reasons: signs of a paper mill; suspected computer-generated content; unreliable results or conclusions; concerns about the data.

We have used six datasets on multifaceted images of X-rays and CT scans. The utilized datasets have been used to evaluate the efficiency of the proposed model compared to the AlexNet, GoogLeNet, and the SVM models. Following comprehensive studies for both datasets of X-rays and CT scans, the proposed model has proved a highly accurate COVID-19 diagnosis. The main contributions of the current study can be summarized as follows to combat COVID-19:

- A review of the state-of-the-art AI solutions.
- Evaluating different AI models for the COVID-19.
- Designing a model for detection and prediction of COVID-19.
- Using six datasets that contained three for the X-ray images and three for the CT images for practical examinations.
- Implementing AlexNet and GoogLeNet models as a pretrained CNN network with the SVM model for the selected datasets.
- Developing a hybrid model for COVID-19 prediction.
- Applying the Friedman test for comparing the proposed models and the different datasets.

The rest of the paper is organized as follows: Section 2 introduces the most recent related works.  Section 3 explains the proposed COVID-19 detection model in detail, and Section 4 illustrates the experimental results and comparisons. Finally, the conclusions and future work are discussed in Section 5.

## 2. Literature Review

With the aid of clinical evidence and chest CT imaging, artificial intelligence (AI) methods could be applied to test the potential risks of critical cases of COVID-19.  Table 1 shows the significant role of technologies that are commonly associated with AI, such as machine learning (ML), deep learning (DL), and neural networks (NN) for COVID-19 detection and diagnosis, classification, and differentiation of this epidemic from other illnesses. DL approaches, including the Convolutional Neural Network (CNN), are recommended to be the appropriate means of achieving the desired targets, especially for COVID-19 prediction and treatments. This is because that form of networks is substantially able of nonlinear modeling and has widespread use in medical image processing and diagnostics [4].

The next section discusses the proposed approach using three standard models with the hybrid ANNBOA model for COVID-19 prediction.

## 3. Proposed COVID-19 Prediction Model

The deep learning approaches have introduced many models in the last two years. In this section, a proposed hybrid model of the butterfly optimization algorithm with the artificial neural network (ANN) is introduced. The proposed model is compared with the pretrained AlexNet, GoogLeNet, and the SVM for diagnosing COVID-19 cases.

There are many advanced improvements for the SVM as in [22–24], but we recommended the standard method for the SVM to show the enhancements of the novel model of the deep learning approaches.  Figure 1 shows the proposed framework for evaluating the ANNBOA, AlexNet, GoogLeNet, and the SVM models for COVID-19 prediction.

The article "Advanced Cognitive Algorithm for Biomedical Data Processing: COVID-19 Pattern Recognition as a Case Study" was retracted in 2023. Reasons: signs of a paper mill; suspected computer-generated content; unreliable results or conclusions; concerns about the data.

The proposed approach can be arranged as follows:

1. Collecting the data using (CT, and X-ray) images.
2. Processing data as resize images, remove noise, normalization, and others.
3. Applying feature extraction using AlexNet, and GoogLeNet models.
4. Classifying the output using the SVM classifier.
5. Developing a hybrid model (BOA + NN).
6. Comparing the hybrid model with the pretrained AlexNet, GoogLeNet, and the SVM.
7. Evaluation and prediction the disease

The proposed approach composed of three layers. The first layer is the dataset collection from different sources of available publicity. The datasets are two categories of the medical images, the X-ray and the CT-scan images.

Datasets considered the essential factor for good training since CNN can learn how to extract significant features from the image and SVM classifier for detection of COVID-19 from these images. The main problem in dataset is the small number of available images about COVID-19 cases nowadays.

The quality of the developed system improves through an effective training process. The trained algorithms are confirmed by three-fold portioning of data (training-testing-validation). The training and testing process in the second layer are the most critical factor in the success of machine learning function. Validation is used to evaluate the performance and maintain the best-trained model for different hyperparameters combinations (e.g., number of iterations, the architecture, and allowable error). A final, unbiased evaluation will be performed on the test set after creating a final model based on training and validation test sets. In this paper, data are divided into training, testing, and validation by a ratio of 5 : 1 : 1, respectively.

By comparing the activated areas of the convolutionary layers with the corresponding regions of the original images, the deep layer features of an image were examined. The activation map can have different values and was thus normalized from 0 to 1. In comparison with the original images, the strongest activation channels from COVID-19 and regular X-ray and CT images were determined. In their first convolutionary layer, convoluted neural networks detect features such as color and edges. The network can see more complicated functions in deeper convolutionary layers. Later, layers create their characteristics by combining features of older layers. COVID-19 could be challenging to distinguish from the original images of various groups of research. However, the deep layer features best explain the reason for the crash or success of a deep learning network in a demanding decision. The third layer is the output layer with the model assessment and non-infection prediction of COVID-19 from infection. Five performance measurements, such as accuracy, sensitivity or recall, specificity, accuracy, and F1 score, assessed the performances of various networks. The proposed model could recognize the X-ray and CT images of COVID-19 from the different datasets, as they present a visual explanation of the CNN and SVM prediction and emphasizes the infected regions, and compare with the proposed hybrid model (BOA + NN) that contribute more to the classification. The proposed ANNBOA model is shown in Figure 2.

The article "Advanced Cognitive Algorithm for Biomedical Data Processing: COVID-19 Pattern Recognition as a Case Study" was retracted in 2023. Reasons: signs of a paper mill; suspected computer-generated content; unreliable results or conclusions; concerns about the data.

As one of the most resilient and effective machine learning approaches, neural networks (NNs) have been widely utilized to solve a variety of issues. However, selecting appropriate parameters (for example, weights) has a major impact on the accuracy of these approaches. As a result, several studies have been conducted to enhance the NN parameters. The training process of artificial neural networks, which is primarily focused on selecting the optimum combination of biases and weights, is one of the most challenging issues in machine learning. Gradient descent techniques are the most widely used training algorithms. They are, nevertheless, vulnerable to local optima and sluggish convergence in training.

The butterfly optimization algorithm (BOA) [25] is a new metaheuristic method that was recently suggested. Its idea comes from the natural food-seeking activity of butterflies. Furthermore, it has been demonstrated that BOA can tackle a wide range of optimization issues and achieving global optimal solutions. A novel classification technique based on the integration of artificial neural networks and the BOA algorithm is presented in this study.

The goal of the backpropagation algorithm (BP) is to improve network parameters by reducing the least square error between actual and calculated output. This section describes the BOA-BP classification technique for training the BP neural network using the BOA. The parameters for the BOA are (*c* = 0.01, a ⟶ [0.1, 0.3], *p*=0.5).

We execute 30 separate training and test runs to achieve significant statistical findings. We used the min-max scaling normalization approach to normalize all of the characteristics of each dataset into the [0, 1] interval, as shown in the following equation:

(1) $$\begin{array}{c} k_{i}^{\prime }=\frac{k_{i\;}-\min_{k}}{\max_{k}-\;\min_{k^{\prime }}}. \end{array}$$

This procedure of normalization is essential before training since it eliminates the influence of one feature having a value in a wider range over another. The pseudocode of butterfly optimization algorithm is shown in Algorithm 1.

The article "Advanced Cognitive Algorithm for Biomedical Data Processing: COVID-19 Pattern Recognition as a Case Study" was retracted in 2023. Reasons: signs of a paper mill; suspected computer-generated content; unreliable results or conclusions; concerns about the data.

Although the suggested strategy has been mainly created for COVID-19 related tasks, it can apply in other medical imaging examinations. Input images are often resized for the convolution network models to maintain network architecture compatibility. The pseudocode of the utilized AlexNet and GoogLeNet models is shown in Algorithm 2.

Because the AlexNet input image is 227 × 227 and the GoogLeNet input image must be 224 × 224, we used the original image set to be redimensionable into two image sets so that both AlexNet and GoogLeNet can be used. Two matrices are necessary to train the SVM. If we have all the extracted features in a single matrix, we have an *N* × *M*, which contains *N* as the image number and *M* as the feature number. The second matrix is a matrix of labels. All image labels in this *N* × 1 matrix are being imported to tell SVM whether the given image from the set is COVID-19 or not. The last input we will use for training the SVM is these two matrices. With the SVM method, we have chosen which features we would like to use and extracted the features with the AlexNet CNN. We can receive features of the images after we have feed images to that layer. We could then use them for training an SVM to detect COVID-19 after all the features are there. The test data are used for model assessment and prediction after training of each model.

## 4. Results and Discussion

In this paper, we attempt to find an SVM, transfer learning and the proposed ANNBOA so that the computers can self-detect if a particular patient is a COVID-19 using CT or X-ray pictures. Softmax was used to classify the fully connected layer with the SVM classifier in the three standard models. The entire experimentation was performed in the 64-bit Windows 10 Pro operating system, Intel(R) 16 GB RAM Core(TM) i7-8550U CPU@ 1.80GHZ 1.99 GHz processor. Each algorithm is used with MATLAB (2018a).

### 4.1. Dataset Description

In this paper, six datasets are used; three for X-ray and three for CT images.  Table 2 gives a brief explanation of the employed datasets.

The total count of the utilized images is 18096 X-ray images, 7406 for COVID-19 cases, and 10690 for normal patients. Also, there are 10977 CT images, 6877 for COVID-19 cases, and 4100 for normal patients. The description of the dataset portioning after removing noisy images is shown in Table 3.

### 4.2. Results

We use a test image set to determine the threshold that can best be accurately determined after the parameters are determined. For CNN, setup is initiated by installing AlexNet and GoogLeNet pretrained networks. A sample of the network training and validation of the accuracy and the error rate (loss) for both AlexNet and GoogLeNet are shown in Figures 3, and 4 respectively.

The article "Advanced Cognitive Algorithm for Biomedical Data Processing: COVID-19 Pattern Recognition as a Case Study" was retracted in 2023. Reasons: signs of a paper mill; suspected computer-generated content; unreliable results or conclusions; concerns about the data.

To evaluate the proposed model, five measures are utilized as follows: accuracy, sensitivity, specificity, precision, and F1 score.

Figures 5 and 6 show the comparison among the different classifiers (SVM, AlexNet, GoogLeNet, and ANNBOA) for the X-ray dataset and CT-scan dataset.

Table 4 shows that all the pretrained models evaluated are successful in classifying COVID-19. SVM, AlexNet, GoogLeNet, and ANNBOA are involved in ranking images among networks trained in different X-ray and CT datasets in the problem of two classes.  Figure 7 shows the mean of performance measurements for the proposed techniques. The results show the superiority of the proposed model (ANNBOA) with average accuracy 90.48%.

### 4.3. Results Discussion

This paper uses deep learning technologies for creating a classification network to distinguish COVID-19 from non-COVID-19 cases. As far as the network structure is concerned, AlexNet, GoogLeNet, and BOA with NN are used to extract features. The experiment showed that COVID-19 cases could be more distinguishable from others by the proposed mechanism. It is noted that from Figure 7 that the BOA with NN achieves the highest results using performance measurements (Accuracy, Sensitivity, Specificity, Precision, and F1-Score). A hypothesis test, called related-samples Friedman's two-way analysis of variance by ranks, is used to compare between proposed techniques in this paper. The null hypothesis is “the distribution of SVM, AlexNet, GoogLeNet, and BOA are the same.” If asymptotic significance is less than the significance level is *α* = 0.05, then the decision is rejecting the null hypothesis. As sown in Table 5, Asymp sig. <0.05, so we reject the null-hypothesis with the mean that there are statistically significant differences between 4 techniques with strong effect according to ES (Effect Size) which is used to detect impact of techniques using the following equation:

(2) $$\begin{array}{c} \text{ES}=\frac{x_{\text{Friedman}}^{2}}{k\left(N-1\right)}, \end{array}$$

as *k* = # measurements, and *N* = # techniques.

The value of ES is compared to the standard values to check the strong of ES. In our case, ES = 0.808 that is between .70 and .90 with strong effects.

Wilcoxon Signed Ranks Test is used to list these statistically significant differences.  Table 6 shows Wilcoxon Signed Ranks test between the proposed techniques. It is noted that there is significant difference between AlexNet and GoogLeNet in favor of AlexNet. Also, there are significant differences between BOA + NN and SVM, AlexNet, GoogLeNet in favor of the BOA + NN technique. So, BOA + NN is the best technique.

The article "Advanced Cognitive Algorithm for Biomedical Data Processing: COVID-19 Pattern Recognition as a Case Study" was retracted in 2023. Reasons: signs of a paper mill; suspected computer-generated content; unreliable results or conclusions; concerns about the data.

The correlations between the BOA + NN and the other techniques, where there are significant differences, are calculated using Spearman's correlation in Table 7.

Figure 8 shows strong positive correlation (*r* = 0.9) between BOA + NN, and SVM as *P* (0.037) < 0.05 in the presence of the five measurement. We conclude from the previous results that BOA + NN technique is correlated with SVM classifiers (positive correlation) to detect disease by high-performance measurements. There are some restrictions in this study; the first thing to do is combines the patient's contact history, travel history, initial symptoms, and laboratory examination with a clinical diagnosis of COVID-19. Second, this study limited the number of model samples. To improve accuracy in the future, the number of training and test samples in the utilized datasets must be extended.

## 5. Conclusion and Future Work

Coronavirus (COVID-19) recently became one of the world's worst and most acute diseases. Therefore, an automated pattern detection system should be used as the fastest possible diagnostic method to prevent the spread of COVID-19. This paper introduced a new approach for automatically screening CT and X-ray images of COVID-19 using deep learning technologies. Models can be classifying different cases for the COVID-19 and non-COVID-19 with the high accuracy among the GoogLeNet, AlexNet, and proposed BOA + NN models in some comparative data sets so that a promising additional diagnostic tool for frontline clinical doctors may be the proposed approach. The findings revealed the dominance of BOA with NN to attain the highest accuracy of all X-ray images. In contrast, in CT images, AlexNet accomplished the highest accuracy in two datasets and GoogLeNet, in one dataset.

In future, we aim to apply different machine learning and deep learning models together with providing strategies to select the most important features using metaheuristic algorithms.

## Figures and Tables

**Figure 1:** Proposed framework for evaluating different models for COVID-19 prediction.

**Figure 2:** Proposed ANNBOA model.

**Figure 3:** Samples from training and validation of AlexNet.

**Figure 4:** Samples from training and validation of GoogLeNet.

**Figure 5:** Comparison among the three classifiers for the X-ray images.

**Figure 6:** Comparison among the three classifiers for the CT-scan.

**Figure 7:** Mean of performance measurements for the proposed techniques.

The article "Advanced Cognitive Algorithm for Biomedical Data Processing: COVID-19 Pattern Recognition as a Case Study" was retracted in 2023. Reasons: signs of a paper mill; suspected computer-generated content; unreliable results or conclusions; concerns about the data.

**Figure 8:** Correlation between BOA + NN and SVM.

**Algorithm 1:** The butterfly optimization algorithm (BOA).

**Algorithm 2:** The AlexNet and GoogLeNet models.

**Table 1:** AI techniques for COVID-19.

Author	Images type	AI methods	Task	Results
Nayak et al. [5]	Chest X-ray (CXR) images	AlexNet, GoogLeNet, MobileNet-V2, SqueezeNet, VGG-16, ResNet-50, ResNet-34, and Inception-V3	Classification of COVID-19 from normal cases	Accuracy of ResNet-34 is 98.33%
Shorfuzzaman and Hossain [6]	CXR images	VGG-16 network	Classification of COVID-19 cases	Accuracy is 95.6% and AUC is 0.97
Linda [7]	CXR images	A deep CNN, namely, COVID-Net	Detection of COVID-19 cases	Accuracy is 92.4%
Rahman et al. [8]	CXR images	Novel U-Net model	Automatic detection of COVID-19	Accuracy is 95.11%
Jin et al. [9]	CT images	2D deep CNN	Rapid COVID-19 detection	Accuracy is 94.98% and AUC is 97.91%
Narin et al. [10]	CXR images	Pretrained ResNet-50	Detection of coronavirus pneumonia-infected patient	Accuracy is 98%
Chowdhury et al. [11]	CXR images	AlexNet, ResNet-18, DenseNet201, and SqueezeNet	Automatic detection of COVID-19 pneumonia	Accuracy is 98.3%
Maghdid et al. [12]	CXR images and CT images	A new CNN and pretrained AlexNet with transfer learning	Effective COVID-19 detection technique	Accuracy is 98% on X-ray images and 94.1% on CT images
Gour and Jain [13]	CXR images	Multiple CNN models	Classification CT samples with COVID-19, influenza viral pneumonia, and no infection.	Accuracy is 96%, sensitivity is 98.2% and specificity is 92.2%.
Kang et al. [14]	CT images	KNN as well as NB	Automatic analysis pipeline for COVID-19	Accuracy 95%, sensitivity 93.2%, specificity 96.6%
Khanday et al. [15]	Clinical data	Multinomial naive bayes and logistic regression	Identifying pandemic with clinical text information	Accuracy is 96.2%
Sethy et al. [16]	CXR images	CNNs with the help of support vector machine (SVM)	Detecting the COVID-19 disease	Accuracy is 95.38%
Alakus and Turkoglu [17]	CXR images	CNN based LSTM, CNN-RNN	Analyzing the COVID-19	Accuracy 86.66%, precision 86.75%, recall 99.42%
Rasheed et al. [18]	CXR images	CNN and logistic regression	Diagnosis of COVID-19	Accuracy is 97.6 for CNN and 100% for LR
Gao et al. [19]	CT images	Dual-branch combination network (DCN)	Accurate diagnosis and lesion segmentation of COVID-19	Accuracy is 96.74% on the internal dataset and 92.87% on the external dataset
Goel et al. [20]	CXR images	Optimized convolutional neural network (OptCoNet)	Automatic diagnosis of COVID-19	Accuracy is 97.78%
Nour et al. [21]	CXR images	SVM	Detection of COVID-19 infection	Accuracy 98.97% sensitivity 89.39% specificity 99.75%

**Table 2:** X-ray and CT-scan for COVID-19 cases and normal cases.

Type	Name	Code	COVID-19	Non COVID-19
X-ray	Extensive COVID-19 X-ray images dataset [26]	DS_1	4044	5500
	Augmented COVID-19 X-ray images dataset [27]	DS_3	912	912
	Combined COVID-19 dataset [28]	DS_5	2450	4278

CT-scan	Extensive COVID-19 CT chest images dataset	DS_2	5427	2628
	SARS-COV-2 Ct-scan dataset [29]	DS_4	1252	1229
	COVID-19 CT scans [30]	DS_6	198	243

The article "Advanced Cognitive Algorithm for Biomedical Data Processing: COVID-19 Pattern Recognition as a Case Study" was retracted in 2023. Reasons: signs of a paper mill; suspected computer-generated content; unreliable results or conclusions; concerns about the data.

**Table 3:** Dataset portioning.

Dataset	COVID-19				Non-COVID-19			
	Training	Validation	Testing	Sum	Training	Validation	Testing	Sum
DS_1	2880	579	575	4034	3822	785	785	5392
DS_2	3701	850	850	5401	1670	475	475	2620
DS_3	650	127	130	907	620	127	130	877
DS_4	895	177	177	1249	845	185	185	1215
DS_5	1378	407	465	2250	2436	715	927	4078
DS_6	132	30	36	198	168	39	36	243

**Table 4:** Output results for SVM, AlexNet, and GoogLeNet.

Dataset	Model	Accuracy	Sensitivity	Specificity	Precision	F1-score
DS_1	SVM	80.96	79.65	81.91	76.33	77.96
DS_2		62.47	71.88	45.78	70.16	71.01
DS_3		**99.23**	99.23	99.23	99.23	99.23
DS_4		83.83	79.44	88.11	86.67	82.90
DS_5		98.94	98.95	98.94	98.21	98.57
DS_6		61.11	100	22.22	56.25	72

DS_1	AlexNet	88.82	92	86.50	83.31	87.44
DS_2		63.94	62.24	67.47	79.83	69.95
DS_3		**100**	100	100	100	100
DS_4		88.21	85.56	90.81	90.06	87.75
DS_5		99	98.50	99.29	98.79	98.64
DS_6		80.56	88.89	72.22	76.19	82.05

DS_1	GoogLeNet	89.12	90.43	88.15	84.83	87.54
DS_2		51.08	45.49	62.67	71.60	55.63
DS_3		**100**	100	100	100	100
DS_4		82.47	79.44	85.41	84.12	81.71
DS_5		99.67	99.55	99.73	99.55	99.55
DS_6		87.5	97.22	77.77	81.40	88.60

DS_1	BOA + NN	91.54	92.35	90.93	88.58	90.42
DS_2		70.46	69.37	71.89	76.39	72.71
DS_3		100.00	100.00	100.00	100.00	100.00
DS_4		89.86	89.82	89.90	88.24	89.02
DS_5		99.72	99.70	99.73	99.55	99.62
DS_6		91.30	97.22	84.85	87.50	92.11

**Table 5:** Friedman test for our proposed techniques.

Model	Mean	Std deviation	Max	Mean rank	Chi-square	Asymp sig.	ES
SVM	81.35	5.63	88.19	1.40	12.12	0.007	0.808 (strong effect)
AlexNet	87.27	0.84	88.03	2.80			
GoogLeNet	85.68	0.74	86.92	1.80			
BOA + NN	90.43	0.70	91.41	4.00			

**Table 6:** Wilcoxon signed ranks test for SVM model.

	AlexNet-SVM	GoogLeNet-SVM	BOA–SVM	GoogLeNet-AlexNet	BOA-AlexNet	BOA-GoogLeNet
Z	−1.753^b^	−1.483^b^	−2.023^b^	−2.023^c^	−2.023^b^	−2.023^b^
Asymp. Sig. (2-Tailed)	0.080	0.138	0.043	0.043	0.043	0.043

b. Based on negative ranks. c. Based on positive ranks.

**Table 7:** Spearman's correlation.

	SVM	AlexNet	GoogLeNet	BOA + NN
SVM				
AlexNet	0.700			
GoogLeNet	−0.200	0.300		
BOA + NN	0.900^*∗*^	0.400	−0.600	

^*∗*^Correlation is significant at the 0.05 level (2-tailed).

## Data Availability

Datasets are publicly archived at https://data.mendeley.com/datasets/8h65ywd2jr/3-https://data.mendeley.com/datasets/2fxz4px6d8/4-https://data.mendeley.com/datasets/3pxjb8knp7/3-https://www.kaggle.com/plameneduardo/sarscov2-ctscan-dataset-https://github.com/UCSD-AI4H/COVID-CT.

The article "Advanced Cognitive Algorithm for Biomedical Data Processing: COVID-19 Pattern Recognition as a Case Study" was retracted in 2023. Reasons: signs of a paper mill; suspected computer-generated content; unreliable results or conclusions; concerns about the data.

## Abbreviations

COVID-19: Coronavirus disease 2019
CXR: Chest X-ray
CT: Computerized tomography
CNN: Convolutional neural network
SVM: Support vector machine
ML: Machine learning
DL: Deep learning
ANN: Artificial neural network.

## References

[1] Singhal T. (2020). A review of coronavirus disease-2019 (COVID-19). *Indian Journal of Pediatrics*.

[2] Nguyen T. T. (2020). Artificial intelligence in the battle against coronavirus (COVID-19): a survey and future research directions. https://arxiv.org/abs/2008.07343.

[3] Allam Z., Jones D. S. On the coronavirus (COVID-19) outbreak and the smart city network: universal data sharing standards coupled with artificial intelligence (AI) to benefit urban health monitoring and management. *Healthcare*.

[4] Hesamian M. H., Jia W., He X., Kennedy P. (2019). Deep learning techniques for medical image segmentation: achievements and challenges. *Journal of Digital Imaging*.

[5] Nayak S. R., Nayak D. R., Sinha U., Arora V., Pachori R. B. (2021). Application of deep learning techniques for detection of COVID-19 cases using chest X-ray images: a comprehensive study. *Biomedical Signal Processing and Control*.

[6] Shorfuzzaman M., Hossain M. S. (2021). MetaCOVID: a Siamese neural network framework with contrastive loss for n-shot diagnosis of COVID-19 patients. *Pattern Recognition*.

[7] Linda W. (2020). COVID-Net: a tailored deep convolutional neural network design for detection of COVID-19 cases from chest radiography images. *Journal of Network and Computer Applications*.

[8] Rahman T., Khandakar A., Qiblawey Y. (2021). Exploring the effect of image enhancement techniques on COVID-19 detection using chest X-ray images. *Computers in Biology and Medicine*.

[9] Jin C., Chen W., Cao Y. (2020). Development and evaluation of an AI system for COVID-19 diagnosis. *medRxiv*.

[10] Narin A., Kaya C., Pamuk Z. (2020). Automatic detection of coronavirus disease (Covid-19) using X-ray images and deep convolutional neural networks. https://arxiv.org/abs/2003.10849.

[11] Chowdhury M. E., Rahman T., Khandakar A. (2020). Can AI help in screening viral and COVID-19 pneumonia?. https://arxiv.org/abs/2003.13145.

[12] Maghdid H. S., Asaad A. T., Ghafoor K. Z., Sadiq A. S., Khan M. K. (2020). Diagnosing COVID-19 pneumonia from X-ray and CT images using deep learning and transfer learning algorithms. https://arxiv.org/abs/2004.00038.

[13] Gour M., Jain S. (2020). Stacked convolutional neural network for diagnosis of Covid-19 disease from X-ray images. https://arxiv.org/abs/2006.13817.

The article "Advanced Cognitive Algorithm for Biomedical Data Processing: COVID-19 Pattern Recognition as a Case Study" was retracted in 2023. Reasons: signs of a paper mill; suspected computer-generated content; unreliable results or conclusions; concerns about the data.

[14] Kang H., Xia L., Yan F. (2020). Diagnosis of coronavirus disease 2019 (COVID-19) with structured latent multi-view representation learning. *IEEE Transactions on Medical Imaging*.

[15] Khanday A. M. U. D., Rabani S. T., Khan Q. R., Rouf N., Mohi Ud Din M. (2020). Machine learning based approaches for detecting COVID-19 using clinical text data. *International Journal on Information Technology*.

[16] Sethy P. K., Behera S. K., Ratha P. K., Biswas P. (2020). Detection of Coronavirus Disease (COVID-19) Based on Deep Features and Support Vector Machine. *Preprints*.

[17] Alakus T. B., Turkoglu I. (2020). Comparison of deep learning approaches to predict COVID-19 infection. *Chaos, Solitons & Fractals*.

[18] Rasheed J., Hameed A. A., Djeddi C., Jamil A., Al-Turjman F. (2021). A machine learning-based framework for diagnosis of COVID-19 from chest X-ray images. *Interdisciplinary Sciences: Computational Life Sciences*.

[19] Gao K., Su J., Jiang Z. (2021). Dual-branch combination network (DCN): towards accurate diagnosis and lesion segmentation of COVID-19 using CT images. *Medical Image Analysis*.

[20] Goel T., Murugan R., Mirjalili S., Chakrabartty D. K. (2021). OptCoNet: an optimized convolutional neural network for an automatic diagnosis of COVID-19. *Applied Intelligence*.

[21] Nour M., Cömert Z., Polat K. (2020). A novel medical diagnosis model for COVID-19 infection detection based on deep features and Bayesian optimization. *Applied Soft Computing*.

[22] Tanveer M., Khan M. A., Ho S.-S. (2016). Robust energy-based least squares twin support vector machines. *Applied Intelligence*.

[23] Tanveer M., Sharma A., Suganthan P. N. (2019). General twin support vector machine with pinball loss function. *Information Sciences*.

[24] Shi Q., Katuwal R., Suganthan P. N., Tanveer M. (2021). Random vector functional link neural network based ensemble deep learning. *Pattern Recognition*.

[25] Arora S., Singh S. (2019). Butterfly optimization algorithm: a novel approach for global optimization. *Soft Computing*.

[26] Walid El-Shafai F. A. E.-S. (2020). *Extensive COVID-19 X-Ray and CT Chest Images Dataset*.

[27] Ali Mohammad Alqudah S. Q. (2020). *Augmented COVID-19 X-ray Images Dataset*.

[28] Fathi Abd El-Samie Ahmed Abd El-Latif Ahmed Sedik M. H. (2020). *Combined COVID-19 Dataset*.

[29] PlamenEduardo (2020). *SARS-COV-2 Ct-Scan Dataset*.

[30] Jkooy S. (2020). *COVID-19 CT Scans*.

